# Genetic Relationship and Evolution Analysis among Malus Mill Plant Populations Based on SCoT Molecular Markers

This article has been retracted.

**DOI:** 10.1155/2022/1002624

**Published:** 2022-06-17

**Authors:** Yuan Yao

**Affiliations:** College of Life Sciences, Shanghai Normal University, Shanghai 200234, China

## Abstract

Malus Mill genotype is highly heterozygous, and many theoretical problems such as genetic relationship and evolution process among germplasm are difficult to be solved by traditional analysis methods. The development of SCoT(start codon targeted polymorphism) molecular markers suitable for apples is of great significance for studying the origin, evolution, genetic relationship and genetic diversity of Malus Mill germplasm resources. In this paper, the genetic relationship and evolution of 15 materials were analyzed by SCoT molecular marker. The results showed that the gene differentiation coefficient values of four Malus Mill plants at the species level were 0.423, 0.439, 0.428 and 0.460, respectively, which indicated that there was obvious genetic differentiation among the populations of these four Malus Mill plants, but there were some differences among the populations of different Malus Mill plants. The gene differentiation coefficient of coextensive populations with different geographical distribution varied from 0.177 to 0.086 (average 0.138), which indicated that the genetic similarity of species in coextensive composite populations was high and there was a close genetic relationship among species. This indicates that SCoT molecular markers can be effectively used in the analysis of intraspecific genetic relationship and identification of intraspecific strains of Malus Mill plants.

## 1. Introduction

Malus Mill is a genus of Rosaceae with high economic value. Malus Mill plants such as M.hallianaKoehne, M.baccata (L.)Borkh, M.hupehensis (Pamp.)Rehd, M.micromalus are important garden trees.Many species are used as rootstocks in apple production [1–3]. The traditional Malus Mill classification is based on botanical characters such as the state of leaves in buds, the whole or shallow split of leaves, the number of styles and the color of stamens, the shedding or persistent sepals, the presence or absence of stone cells in pulp, and experimental taxonomic evidence such as chromosomes, plant chemical components and isozymes. Based on the development of molecular technology in recent years, it has become the mainstream to use molecular marker technology to reveal the genetic relationship between apple germplasm resources and materials, analyze the differences among materials from the genome level, and then assist breeders to choose suitable combinations of apple hybrid parents [4–6] However, the genomic sites revealed by different markers are different, and the sequence information that can reveal the different sites may not be transcribed and expressed.

Genetic marker is an easily recognizable manifestation of biological genotype. With the understanding of gene from phenomenon to essence, genetic marker has gradually developed from simple morphological marker, cytological marker and biochemical marker to DNA molecular marker which can directly reflect genetic polymorphism at the DNA level [7].Scot (start codon targeted polymorphism) marker is a new marker method created by Collard and others in rice. This marker is not only highly polymorphic, but also convenient to operate. At present, it has been applied to the research of many fruit trees and plants. In addition, there are markers that use specific double primers to amplify and analyze the polymorphism of specific DNA regions, mainly including AFLP (amplified fragment length polymorphism), SCAR (sequence characterized amplified regions) and STS(Sequence Tag Site), among which AFLP markers are widely used. SCoT marker has been successfully applied to citrus [8], Dendrobium candidum and other crops [9, 10], and much progress has been made in the research of genetic diversity among species and varieties and genetic analysis of hybrid offspring. With more and more evidences being introduced into the systematic study of this genus, for example, whether the calyx of fruit persists, the growth state of leaves in buds, whether the fruit has stone cells or not, and the experimental new classification system such as chromosomes, plant chemical components, enzymes, molecular biology, etc., are more scientific, which can better reflect the genetic relationship and evolution path among plant groups in this genus.

The emergence and development of DNA molecular markers make molecular systematics one of the latest experimental classification methods, and SSR (simple sequence repeats) markers with unique advantages have been widely used in Apple research [11, 12].However, the development of traditional genomic SSR markers needs complicated steps such as constructing genomic DNA library, probe hybridization, cloning and sequencing [13], which is time-consuming, labor-intensive and costly. The application of SSR markers is greatly limited. As a new SSR marker, SCoT marker has been applied in many plants such as grape, sugar cane, wheat, barley, soybean, rice and other species such as genetic diversity analysis, genetic map construction and systematic evolution research [14, 15]. Research on systematic classification and genetic relationship of apple cultivars based on SCoT technology has not been reported. In this study, making full use of database resources and developing new SCoT markers from Malus MillEST database will not only further enrich the number of markers, but also provide a new way for the study of genetic relationship of this genus.

## 2. Related Work

SCoT marker can not only obtain the target genes closely related to traits, but also track traits. It has the advantages of simple operation, high polymorphism, abundant genetic information, low cost and strong universality of primers, among which the most prominent ones are high polymorphism detection efficiency and abundant genetic information. At present, it has been widely used in the research of genetic diversity, population genetic structure, germplasm identification, gene differential expression and molecular genetic map of plant germplasm resources. Literature [16] Construction of DNA fingerprint of Hemarthria spp cultivated plants by EST-SSR and SCoT markers; Literature [17] The application of SCoT molecular marker correspondence in the genetic analysis of Nicotiana plants and the identification of interspecific hybrids found that SCoT-labeled primers can be used for the analysis of the genetic relationship between tobacco species and the identification of distant hybrids. Literature [18] used SCoT diversity marker to mark the difference of genetic diversity between wild and cultivated species of Boehmerianivea L. Gaudich; Literature [19] The application of SCoT molecular marker correspondence in the genetic analysis of Nicotiana plants and the identification of interspecific hybrids found that SCoT-labeled primers can be used for the analysis of the genetic relationship between tobacco species and the identification of distant hybrids. At present, the application of this technology in medicinal plants has been reported.

Genetic diversity refers to the sum total of genetic variation among different groups or individuals within a group, which is the basis and important component of biodiversity. The evaluation of genetic diversity of plant natural populations and artificially cultivated strains is the basis of effective protection, development and utilization of germplasm resources. Literature [20] 100 pairs of SSR primers were developed and designed from EST database of citrus to detect the genetic diversity and heterozygosity of two different citrus genera, Citrus sinensis(L.)Osbesk and Poncirus trifoliate(L.)Raf. Literature [21] Sixteen pairs of SSR primers were selected and designed from EST of grape to detect the genetic diversity of seven grape varieties, among which 10 pairs of primers could amplify polymorphic bands in these tested materials. Literature [22] Through cluster analysis, it is shown that Chinese varieties and other varieties in the world are clustered into two separate groups, respectively, while the hybrids of two peaches and apricots are closer to peaches in genetic relationship, and they are clustered into an outer group together. Literature [23] The genetic relationship among wild apples, cultivated apples and ornamental begonia originated in Belgium and Germany was analyzed by AFLP and SSR. Literature [24] also used SSR and SRAP markers to analyze the genetic relationship of apples. In this study, AFLP, SSR and two molecular markers were used to study the genetic relationship among 41 Malus Mill plant types, and the differences between the two techniques were discussed, which provided reference for the application of AFLP and SSR in the genetic relationship analysis of apples. Literature [25] RAPD (Random Amplified Polymorphic DNA) technology was applied to study the genetic relationship of Malus Mill plants, and the results were basically consistent with previous studies. However, in this study, only 10 primers were screened. For Malus Mill plants with complex origin and evolution, the results only have reference value, and cannot fundamentally solve our questions. Literature [26] AFLP technology has been applied to the study of the relationship between Malus Mill plants, and most of the classification results are the same as those of previous studies. Although this method is accurate, it is only for reference, and it still needs to be combined with other research results. Literature [27] expounds the practical value of M.hupehensis (Pamp.)Rehd. Compared with several other Malus Mill plants with apomixis, M.hupehensis (Pamp.)Rehd has the strongest apomixis ability. The results of SSR molecular markers of M.baccata (L.)Borkh in literature [28] showed that all materials had high genetic diversity, among which M.baccata (L.)Borkh from Hebei had the highest genetic diversity.

Malus Mill, as a classified “difficult genus”, is characterized by diverse plant forms, complex variation of characters, and the intersection of characters among many species is difficult to classify. Due to the widespread interspecific hybridization, many species have complicated classification problems, which are difficult to identify. Literature [29] holds that M.hupehensis (Pamp.)Rehd should be tied to M.baccata (L.)Borkh, while literature [30] holds that M.hupehensis (Pamp.)Rehd should be incorporated into M.baccata (L.)Borkh as a species. More powerful evidence is still needed to prove this. M.hupehensis Rehd. var.taiensis and M.hupehensis (Pamp.)Rehd.var. Mengshanens are two varieties of M. Hupehensis (Pamp.) Rehd, and they also need a strong evidence to prove their relationship with each other and with M. Hupehensis (Pamp.) Rehd.var. Mengshanens. Literature [31] holds that M.hupehensis (Pamp.)Rehd is a multi-point origin, but its origin mechanism has not been determined. The wide application of molecular marker technology has brought us hope to solve the problem. Compared with other technologies, this technology is expressed in the form of DNA, which has higher polymorphism and is not restricted by the environment. However, only using primers to amplify some small fragments of DNA for cluster analysis can only find the genetic diversity, and cannot provide strong evidence for judging the genetic relationship between species. A large number of studies also show that this technology can not fundamentally solve this problem.

Gene mapping is an important condition for obtaining excellent genes. When new genes appear in genetic breeding work, it is necessary to locate them on specific chromosomes, and measure their arrangement order and distance on chromosomes, so as to quickly and accurately locate genes. The key of gene mapping is to determine the parent combination between the populations used for mapping. Molecular markers play an important role in the germplasm resources of fruit trees. Molecular markers have many advantages, such as greatly improving the efficiency of animal and plant varieties, helping to develop and identify new varieties, and reducing breeding costs through marker-assisted breeding. Developing more new molecular markers is the new direction of molecular marker technology development in the future, and it is also the effort direction of researchers. In-depth research on fruit tree germplasm resources by molecular markers is beneficial to all fields, which has become an irreversible trend.

## 3. Research Method

### 3.1. Materials and Methods

#### 3.1.1. Material

The materials used are M.hupehensis (Pamp.)Rehd.var. Mengshanens, M. Hupehensis (Pamp.) Rehd, M.hupehensis Rehd. var.taiensis, M.toringo De Vriese, M.toringoides(Rehd.) Hughes, M.sikkimensis (Wenz.)Koehne, Riwacrabapple, M.rockii Rehder. The collected Malus Mill fruits are mashed and washed with water to separate the seeds from the pulp, dried to remove impurities, and the complete and full seeds are selected and stored in a refrigerator at 4°C for later use.

The treated seeds were put into a refrigerator at 4°C to break dormancy at low temperature, and after 21 days, the seeds were put into an incubator at 28°C. Cross experiments were conducted on the time of breaking dormancy and the optimum temperature for seed germination after breaking dormancy. It was found that the dormancy of seeds could be basically broken in about 21 days, and 28°C was the optimum temperature for seed germination, and the time of breaking dormancy of different species was slightly different.

ProFlex™ PCR System PCR thermal cycler, MultifugeX1R high-speed freezing centrifuge, Gel Doc™ EZ gel imaging system, JY600C electrophoresis tank, Thermo Scientific Nano-Drop 2000 Spectrophotometers spectrophotometer.

Among the published SCoT primers of Malus Mill plants, the primers with high polymorphism and good stability were selected for the experiment. Among the SCoT-labeled primers, three fluorescent markers FAM (6-carboxy-fluoroscein,), hex (hexachlorofluoroscein) and Tamra (carboxy tetramethylrhodamine) were added to the 5' end of each pair of primers.

### 3.2. Method

#### 3.2.1. Extraction and Concentration Determination of DNA

The total DNA of apple leaves was extracted by improved CTAB (cetyltrimethylamine bromide) (Figure 1):

1. Put an appropriate amount of apple leaves in a mortar, add a small amount of quartz sand, grind into powder, and subpackage into 1.5 mLeppendorf tubes
2. Cells were lysed for 30 min~60 min in the warm bath of 65°C constant temperature water bath pot, during which the centrifugal tube was turned upside down for 2 ~ 3 times
3. Suck the supernatant, add 1/10 times the volume of 3mm · L^‐1^Na Ac and 2 ~ 2.5 times the volume of frozen absolute ethanol, and mix carefully
4. Put it in the refrigerator at-20°C for 30 min, gently pick out the flocculent precipitate in the tube, and put it into a new centrifuge tube (or centrifuge at 12000 rpm for 15 min, and pour out the supernatant).
5. Dry DNA at room temperature, add 1 × TE 5 *μ*L dissolved DNA in EP tube, add 1 *μ*L RNase, and keep at 37°C for 1 h or -4°C for one night
6. The extracted DNA was stored in a refrigerator at -20°C

The extracted DNA was detected by 1% agarose gel electrophoresis. The DNA with high brightness, clear main band and no dispersion band was diluted and put into the ultraviolet spectrophotometer for detection. The ratio of OD260/280 was between 1.7 and 1.8, and the purity was high. The DNA concentration was calculated by probe labeling, and the concentration of DNA sample (*μ*g · *μ*L^‐1^) = OD260×50× dilution multiple×1000.

#### 3.2.2. SCoT-PCR Amplification Procedure and Product Detection

Each organism has a specific chromosome number, so it is particularly important to choose appropriate materials to count the chromosome number. Literature [26] holds that the development trend of angiosperm karyotype is from symmetry to asymmetry. That is to say, the karyotypes of plants that are in a relatively primitive taxonomic position in systematic evolution are mostly symmetrical; The karyotype of relatively more evolved plants is mainly asymmetric.

There are still the following scientific problems to be solved in research:

1. The level of genetic diversity in Malus Mill plants and its formation reasons
2. The degree and direction of interspecific hybridization and infiltration of coextensive species and its influence on species formation and differentiation
3. The origin of Malus Mill plant hybridization and the revelation of the “identity” of hybridization, and the reasons for the differences of Malus Mill plant populations distributed in foreign countries

The above research will provide favorable evidence for revealing the mechanism of species formation and evolution of Malus Mill. The technical route is shown in Figure 2:

The PCR amplification reaction system was improved on the basis of the optimized system obtained in reference [22], and the final reaction system was determined as follows: Premix Tap™10 *μ*L, DNA template 2 *μ*L, primer 2 *μ*L, and finally ddH_2_O was added, with a total volume of 20 *μ*L L.

Then, it was placed in a PCR instrument for amplification reaction, and the amplification procedure was pre-denaturation at 94°C for 3 min. Denaturation at 94°C for 30 s, annealing at 55°C for 30 s, renaturation at 72°C for 1 min, 33 cycles; Finally, 72°C for 5 min.

After the PCR amplification procedure is completed, 5 ~ 8 *μ*L of amplification products are slowly dropped into 1% agarose gel with nucleic acid dye, then placed in electrophoresis tank without electrophoresis in electrode buffer (1 × TAE) for 30 min, and then images are collected and saved by gel imaging system.

#### 3.2.3. Data Processing

Image Lab(BIO-RAD) is used to analyze the film, and the number of DNA bands amplified by each treatment is counted. After manual correction, D2000 DNA Marker is used as the reference standard molecular weight to predict the molecular weight of amplified bands, and the molecular weight is regarded as the same position within the range of 5 BP. Then, statistics are made according to the size and site of amplified fragments of each sample. The number of bands at the same position is “1”, and the number of bands with no bands or weak bands that are difficult to distinguish at the same position is “0”.

Then, the similarity coefficient is calculated by the Qualitative date program in NTSYS-pc2.10e data software, and the similarity coefficient matrix is obtained. The SHAN program and UPGMA method are used for cluster analysis, and then the cluster diagram is generated by Treeplot module.

## 4. Results Analysis and Discussion

### 4.1. Genetic Relationship and Its Evolution Results

The successful preparation of DNA and the avoidance of partial degradation are the basis and key to the success of SCoT, because the quality of the template, that is, whether it contains polysaccharides, polyphenols, protein, quinones and pigments, will affect the future PCR amplification reaction. In this experiment, the improved CTAB method was used to extract apple genomic DNA, and the OD260/OD280 values of the tested materials were all between 1.8 and 2.0. 0.8% agarose gel electrophoresis showed that the main band was clear, without degradation, and the purity was high, which met the requirements of SSR analysis.

The most amplified bands of 9 SCoT primers were SCoT12, with 1,344 bands, and the least was SCoT9, with 688 bands. The average number of amplified bands per primer was 948.The polymorphism ratio of 9 primers ranged from 72.5% to 100%, among which SCoT33 had the highest polymorphism ratio and SCoT12 had the lowest polymorphism ratio, and the average polymorphism ratio (Np) of 9 SCoT primers was 85.34%. The polymorphism ratio of each primer is shown in Figure 3.

Malus Mill plant seeds have dormancy phenomenon, so it is the most important step to explore the conditions for breaking seed dormancy to obtain experimental materials. The fifteen Malus Mill plant experimental materials studied in this experiment include eleven wild species materials (M.hupehensis (Pamp.) Rehd. var.Mengshanens), M.hupehensis Rehd. var.taiensis, M.hupehensis (Pamp.)Rehd, M.baccata (L.)Borkh, M.rockii Rehder, M.dumeri (Bois.)Chev, M.toringoDe Vriese, M.toringoides(Rehd.) Hughes, M.sikkimensis (Wenz.)Koehne, Riwacrabapple, M. ombrophila Hand.-Mazz) and four cultivar materials (M. ×robusta Rehd, M. micromalus Makino, M. purpurea, M. ‘Donghongguo').

According to the degree of chromosomal evolution, most of Malus Mill plants in this study are metaphase chromosomes and near metaphase chromosomes, with a karyotype of 2B, which belongs to a relatively primitive type. The karyotype of M.ombrophilaHand-Mazz is 1A, the most primitive, and that of M.toringo De Vriese is 3B, the most evolutionary.

Karyotype parameters of fifteen Malus Mill taxa are shown in Figure 4. The number of hybridized chromosomes and the proportion of hybridized chromosomes between each probe and the test material are shown in Figure 5 (A, B and C, respectively, represent M.hupehensis (Pamp.)Rehd.var. Mengshanens as probe, M. Hupehensis (Pamp.) rehd as probe and M.hupehensis Rehd. var.taiensis as probe).

According to the number of hybrid chromosomes, the chromosome homology between them is lower than that of M.toringo De Vriese and M.toringoides(Rehd.) Hughes, that is, the genetic relationship between them is not high. In the next research, the screening range of parents of M.hupehensis Rehd. var.taiensis should be expanded.

### 4.2. Genetic Structure of Malus Mill Natural Population

According to Nei's gene diversity analysis, the gene differentiation coefficient values of four Malus Mill plant species at the level of M. baccata(L.) Borkh, M.rockii Rehder, M.doumeri (Bois.)Chev. and M. Toringo de Vriese were 0.423, 0.439 and 0.428, respectively. 0.460, indicating that there is obvious genetic differentiation among the populations of these four Malus Mill plants, but there are some differences in the degree of population differentiation among different Malus Mill plants. That is, the main source of intraspecific genetic variation of four Malus Mill plants is intra-population variation among individuals, and the intraspecific genetic differentiation has reached a very significant level (P <0.001). As shown in Table 1.

In order to further explore the relationship between genetic distance and geographical distance, Mantel tests were carried out on the genetic distance and geographical distance of four tested species (Figure 6). The results showed that the genetic distance and geographical distance of four Malus Mill plants were significantly correlated.

Cluster results of 15 materials by principal coordinate analysis (Figure 7).

It was found that 15 test materials were divided into three categories. Three species of Pyrus are the first category; M. doumeri (Bois.) of Malus mill Chev, grassland Begonia and narrow leaf Begonia are the second category, among which grassland Begonia and narrow leaf Begonia are more closely related. The third category is divided into four sub groups. The first category includes Hawthorn Begonia and m. ombrophila hand- Mazz and Dianchi Begonia, M. ombrophila hand- Mazz is closely related to Begonia Dianchi;

Category 2 includes M. sikkimensis (Wenz.) Koehne, M.toringoides(Rehd.) Hughes and begonia; The fourth category includes: M. halliana Koehne, Xinjiang wild apple, betel seed, catalpa seed, flat edge Begonia, Chinese apple, Oriental apple, forest apple and brown Begonia.

The analysis of population structure of 15 tested materials by using Structure 2.3.1 software showed that the number of allele frequency characteristic types K in the samples showed a continuous increasing trend. When K =3, from the distribution of the maximum covariant Q value of 15 materials, the covariant Q of 13 materials is ≥0.6, accounting for 69.7% of the tested materials, indicating that the genetic relationship among these materials is single (Figure 8).

The composite ratio and efficacy index can evaluate the efficiency of marker polymorphic sites and the efficiency of site polymorphism (Figure 9). Among them, ANEA: average effective allele number, AEHL: average expected heterozygosity of locus.

Among the two markers, the effective recombination ratio and efficacy index of ScoT are higher than those of EST-SSR, and SCoT marker has higher polymorphism detection efficiency. The marker index can comprehensively reflect the expected heterozygosity and effective recombination ratio of the average locus. The SCoT marker is 2.337, which is higher than the EST-SSR marker of 1.199.

### 4.3. The Interspecific Genetic Relationship of Apple Genus Coextensive Population

In order to study whether there is mutual influence of population genetic structure among the sympatrically distributed species of Malus, this experiment analyzed the genetic structure of apple species within four sympatrically distributed populations of Malus, namely populations A, B, C and D (Table 2).

The results showed that the gene differentiation coefficient of coextensive populations with different geographical distribution varied from 0.177 to 0.086 (average 0.138), which indicated that the genetic similarity of species in coextensive composite populations was high and there was a close genetic relationship among species. The average gene flow among individuals in the same domain distribution population is 3.362, which indicates that the frequency of gene exchange among several species of Glycyrrhiza uralensis Fisch. distributed in the same domain is higher.

However, the degree of interspecific differentiation in coextensive populations in different regions is relatively different, and the degree of genetic differentiation among species in group A is the highest, which indicates that there are differences in the degree of gene exchange among species in coextensive populations in different regions. The more frequent the gene exchange, the higher the genetic similarity among species. It shows that there are differences in the degree of inter-species gene exchange among coextensive populations in different regions. The more frequent the gene exchange, the higher the genetic similarity among species.

### 4.4. Discussion

Malus Mill plants have natural hybridization [10]; The existence of hybrids in wild environment and different types of variation within species makes the classification and identification based on morphology complicated [20]. The pod shape of some wild apples is a transitional type between two or more apples, or it is inclined to one kind, such as Malus Mill plant group, which makes it difficult to classify and identify species, so it is necessary to classify and identify species by molecular markers.

Among the designed 35 pairs of primers, 16 pairs can amplify polymorphic products. The reason why some primers cannot amplify products may be [10]: The primer sequence falls on two exons; There is a long intron between the two primers, and no product can be amplified. Wrong sequence information was used in primer design. When there are multiple alleles in the analyzed materials, although their coding regions and functions are the same, but the DNA sequences are not completely the same, the amplified products may have fragments with different sizes than expected. The specificity of the primer itself is not high enough to amplify the sequence homologous to the primer.

The results of population structure analysis are also consistent with the results of cluster analysis and principal coordinate analysis. SCoT, IRAP and SSR all divide apple species into three groups when K =3, one of which is Malus Mill plant materials in North China and Northwest China, the other is Malus Mill plant materials in East China and South China, and the last is Malus Mill plant materials in Southwest China. From their structural analysis chart, it can be found that most apple varieties have gene exchange, and Malus Mill plants with similar regions are more likely to have gene exchange, which indicates that whether Malus Mill plant populations are hybridized or not is related to their regional distribution.

The results are the same as those obtained by AMOVA analysis (Table 1) that only a small part of the variation of four Malus plants comes from among populations. According to the traditional concept of gene flow, gene flow can prevent population differentiation caused by local adaptation or genetic drift. The gene flow among four species of Malus plants is less than 1, and there may be some obstacles in gene communication among populations due to geographical isolation effect.

According to the analysis of gene differentiation coefficient, the genetic similarity among the four coextensive populations is high, and the gene flow among the coextensive populations is higher than that among the intraspecific populations. In addition, the analysis of the genetic distance among the coextensive composite populations (Table 2) shows that the genetic distance among the species within the populations is small, and the individual clustering is always the priority clustering of coextensive species, which indicates that the gene flow among coextensive species is caused by hybridization. In addition, during the continuous interspecific hybridization and backcross in this population, new homozygous individuals of genetic type also appeared, such as M.doumeri (Bois.)Chev with homozygous genetic background in the subgroup, which also means that interspecific hybridization of Malus may lead to the formation of new species.

Karyotype analysis and genome in situ hybridization both showed that Malus Mill's plant classification system still had some imperfections.M.hupehensis Rehd. var.taiensis and M.hupehensis (Pamp.)Rehd.var. mengshanens are both variants of M. hupehensis (Pamp.) rehd. The number of chromosomes with hybridization signals is less than that of M.toringo De Vriese and M.toringoides(Rehd.) Hughes, The number and proportion of chromosomes with hybridization signals in M.sikkimensis (Wenz.)Koehne, M.toringoides(Rehd.) Hughes and M.toringo De Vriese are also higher than those in M. M.hupehensis Rehd. var.taiensis, so it is necessary to further study the genetic relationship among Malus Mill plants.

In this experiment, the results obtained by cluster analysis, principal coordinate analysis and population structure analysis are roughly the same, and all three methods effectively show the genetic relationship and genetic diversity among Malus Mill materials. However, there are obvious differences in the classification order of groups and lines, which may be related to the fact that Malus Mill plants have both wild species and cultivated species, and there are many interspecific hybrids. There may be some differences between genetic relationship analysis at molecular level and morphological genetic relationship analysis based on some characters, and there may also be differences between different molecular marker techniques.Literature [26] studies the genetic diversity of apple male resources by means of cluster analysis and principal coordinate analysis, effectively distinguishing apple interspecific resources from different regions. Literature [13] makes population structure analysis and principal coordinate analysis of 146 Malus Mill materials, which can well reveal their genetic relationship and genetic diversity. It can be seen that principal coordinate analysis, cluster analysis and population structure analysis are effective and reliable for identifying the genetic relationship of Malus Mill plants.

To sum up, Malus Mill plants in its neighborhood and coextensive distribution area, the transitional hybridization zone formed by interspecies hybridization, on the one hand, provides a source of variation for species evolution; On the other hand, Malus Mill plants in the hybridization zone, as an interspecific transition group, become the medium of gene flow among Malus Mill plants, and accelerate the gene exchange among Malus Mill plants. It is speculated that in the evolution process of Malus Mill plant species, due to the imperfect reproductive isolation mechanism, there has been a certain inter-species gene exchange. The evolution and formation of Malus Mill plants are related to the parent species with the same domain and domain distribution, which is more in line with the neighborhood and same domain model [16].

## 5. Conclusion

In this study, SCoT molecular markers were used to study the genetic relationship among Malus populations, and the influence of interspecific hybridization infiltration on species formation and differentiation was discussed, and the formation and evolution trend of hybrid Malus plants was analyzed. The main conclusions are as follows:

SCoT marker has a high polymorphism and a large amount of information, which can reveal the level of genetic diversity and genetic relationship between Malus Mill plants and within species. It is an effective molecular marker for studying the genetic structure of Malus Mill natural population, interspecific gene infiltration and so on.

It is proved that M.sikkimensis (Wenz.)Koehne and M.toringoides(Rehd.) Hughes are closely related to M.baccata (L.)Borkh group. M.hupehensis Rehd. var.taiensis and M.hupehensis (Pamp.)Rehd.var. mengshanens are the same varieties of M. hupehensis (Pamp.) rehd. Although the chromosome homology is not high, their morphology is similar. Riwacrabapple is quite different from M.sikkimensis (Wenz.)Koehne, which supports its independent seed formation; Support the viewpoint of M.hupehensis (Pamp.)Rehd's multi-point origin.

The diversity level of Malus plants is higher than that of other apple species distributed in the same domain, and it has certain advantages in quantity and adaptability, which promotes gene exchange among Malus plants.

The classification system and genetic relationship of Malus Mill plants are becoming more and more clear, but the intra-genus classification system needs further improvement, and the inter-species and intra-species relationships need further experiments to prove that the classification of Malus Mill plants still needs further study.

## Figures and Tables

**Figure 1:** Process of extracting total DNA from apple leaves.

**Figure 2:** Technology roadmap.

**Figure 3:** SCoT polymorphism analysis.

**Figure 4:** Karyotype parameters of fifteen Malus Mill taxa.

**Figure 5:** Experimental results of genomic in situ hybridization.

**Figure 6:** Mantel detection of correlation between geographical distance and genetic distance.

**Figure 7:** Principal coordinate cluster analysis of 15 Malus Mill and Pyrus materials.

**Figure 8:** The distribution of the maximum Q value of all kinds of groups in mathematical model.

**Figure 9:** Marking efficiency analysis.

**Table 1:** Genetic structure variance analysis.

Species	Source of variation	Degree of freedom	Variance	Mean square deviation	Variance component	Percentage variation (%)	P-value
M. baccata(L.) Borkh	Intergroup	10	1436.22	133.02	17.26	30	<0.001
	Within population	44	2088.17	44.17	40.06	70	

M.rockii Rehder	Intergroup	5	566.13	146.39	20.36	33	<0.001
	Within population	20	876.91	30.35	40.01	67	

M.doumeri (bois.)Chev.	Intergroup	9	1066.87	128.16	41.33	20	<0.001
	Within population	41	2869.32	40.27	27.69	80	

M.toringo De Vriese	Intergroup	10	1102.75	133.69	16.87	46	<0.001
	Within population	44	2126.82	46.75	33.21	54	

**Table 2:** Population genetic distance.

Group A	Species	M. baccata(L.) Borkh	M.rockii Rehder	M.doumeri (bois.)Chev	
	M. Baccata(L.) Borkh	—	—	—	
	M.rockii Rehder	0.096	—	—	
	M.doumeri (bois.)Chev	0.052	0.055	—	

Group B	Species	M. baccata(L.) Borkh	M.rockii Rehder	M.doumeri (bois.)Chev	M.toringo De Vriese
	M. Baccata(L.) Borkh	—	—	—	—
	M.rockii Rehder	0.093	—	—	—
	M.doumeri (bois.)Chev	0.046	0.042	—	—
	M.toringo De Vriese	0.033	0.049	0.013	—

Group C	Species	M. baccata(L.) Borkh	M.rockii Rehder	M.doumeri (bois.)Chev	
	M. Baccata(L.) Borkh	—	—	—	—
	M.rockii Rehder	0.022	—	—	—
	M.doumeri (bois.)Chev	0.026	0.021	—	—

Group D	Species	M. baccata(L.) Borkh	M.rockii Rehder	M.doumeri (bois.)Chev	M.toringo De Vriese
	M. Baccata(L.) Borkh	—	—	—	—
	M.rockii Rehder	0.103	—	—	—
	M.doumeri (bois.)Chev	0.168	0.027	—	—
	M.toringo De Vriese	0.144	0.026	0.026	—

## Data Availability

The labeled dataset used to support the findings of this study are available from the corresponding author upon request.
